# Establishment of a Big Data Monitoring Platform for Cinema Opening in the Postepidemic Era from the Perspective of Public Health

**DOI:** 10.1155/2022/6505990

**Published:** 2022-08-09

**Authors:** Qi Wei, Nan Zhao

**Affiliations:** ^1^Henan Normal University, Xinxiang 453000, Henan, China; ^2^Yantai University, Yantai 264000, Shandong, China

## Abstract

The emergence of COVID-19 has had a huge impact on people's lives around the world. With the vaccine and the effective policies of the government, the spread of the epidemic has been effectively contained. However, in the postepidemic era, public health and epidemic protection policies have forced the transformation of public places such as movie theaters. The cinema box office monitored by the traditional monitoring platform can no longer effectively reflect the opening of the transformed cinema. To make up for the shortcomings of the traditional monitoring platform, considering the large amount of data generated by the cinemas' online and offline platforms and public place codes, this study establishes an intelligent monitoring platform based on big data technology to monitor the opening of cinemas. The established intelligent monitoring platform can fully extract the feature information contained in numerous data collected from cinemas and output quantitative indicators that characterize the opening of cinemas based on the feature information. The performance of the established intelligent monitoring platform is analyzed through a case study. The research results show that the average relative error between the cinema opening indicators predicted by the intelligent monitoring platform and the real results is within 2%, which indicates that the intelligent monitoring platform has good prediction accuracy. In addition, the statistical analysis results show that the linear correlation coefficient between the predicted and real results is 0.9802 > 0.95, which further indicates the feasibility of the established intelligent monitoring platform to monitor the opening of cinemas in the postepidemic era.

## 1. Introduction

Since 2019, the sudden arrival of coronavirus disease 2019 (COVID-19) has disrupted people's daily life [1]. Due to the rapid spread of COVID-19 and the great threat to people's health, various measures have been taken around the world to deal with the impact of COVID-19. In the background of the COVID-19 pandemic, politics, economy, and life around the world have been widely affected [2, 3]. In terms of politics, to curb the spread of the epidemic, policy responses have been introduced around the world, and protective measures such as vaccination, health code inquiry, and patient isolation and treatment have been adopted [4, 5]. These measures have increased the burden on the government and consumed a lot of manpower, material, and financial resources. On the economic front, due to the impact of the epidemic, stores, enterprises, and other offline units cannot carry out normal work and are facing bankruptcy. At the same time, the reduction of offline consumption has greatly affected the normal operation of the national economy. In terms of life, under the influence of the epidemic, public places cannot be opened normally, and large-scale events cannot be held normally, which makes people's spiritual needs unmet. In addition, due to the need for epidemic prevention and control, people's daily travel and shopping also have many inconveniences [6].

As a public place that provides leisure and entertainment, cinemas are also inevitably affected by the epidemic. During the rapid spread of the epidemic, the government issued strict epidemic prevention and control policies, which forced the cinema market in various places to be suspended. At the same time, under the influence of the epidemic, many completed films were forced to withdraw because they could not be shown. This has impacted the capital chain of the film industry, making it impossible for subsequent projects to proceed smoothly. Due to the failure of the film production and the inability of the film to play normally, the film inventory is insufficient, which affects the subsequent broadcast of new episodes, leads to the cancellation of film-related publicity activities, and the inability of the project to proceed smoothly, etc., which will give film and television companies a series of chain reactions. Fortunately, with the development of vaccines and the effective implementation of epidemic prevention measures, the epidemic has been effectively contained [7, 8]. To improve people's quality of life, various public places such as cinemas have also been reopened. However, although cinemas have been reopened, their operating order is still affected by the epidemic prevention and control policies. In this study, we refer to the era when cinemas and other public places can open in an orderly manner as the postepidemic era.

In the postepidemic era, to provide people with leisure and entertainment while consolidating the public health protection network, cinemas have adopted a series of epidemic prevention and control measures. For example, formulate an emergency response plan for the epidemic and report abnormal situations promptly; reserve e-tickets online to reduce direct contact, and the attendance rate for each show does not exceed 75%; strictly enforce temperature checks; stages are staggered between halls to reduce audience gatherings. To maintain income in the postepidemic era, cinemas have increased the opening of supporting industries. For example, new formats such as trendy games, script killing, and immersive entertainment have been introduced into the cinema space; in addition, to maximize the place effect of cinemas, the development of multifunctional cinema complexes is also a current development trend. Cinema complexes centered on movie content can satisfy the interests of various groups of people, thereby attracting more consumers. Therefore, according to the above analysis, in the postepidemic era, the opening model of cinemas has changed to a certain extent compared with the traditional cinema opening model. To monitor the opening of cinemas in the postepidemic era, it is necessary to monitor not only traditional indicators such as cinema opening rates and box office revenue but also people flow indicators in cinemas. The monitored people flow indicator not only reflects the number of people watching a movie but can also reflect the number of people consuming other entertainment items in the cinema complex [9].

Currently, traditional cinema data monitoring platforms usually monitor the opening of cinemas by summarizing data from ticketing software and offline sales front desks. This traditional monitoring platform can effectively reflect the opening and revenue of cinemas without the impact of the epidemic. However, the transformation of cinemas in the postepidemic era makes this traditional monitoring platform limited in monitoring the flow of people in new entertainment projects. In addition, this traditional monitoring platform does not consider the impact of public health protection policies on the opening of movie theaters. Therefore, to cope with the limitations of traditional cinema data monitoring platforms in the postepidemic era, this study introduced big data technology to build an intelligent cinema opening monitoring platform. Compared with the traditional monitoring platform, the intelligent monitoring platform based on big data technology can make full use of the large amount of data information generated by the Internet platform [10] and extract the feature information that characterizes the opening of the cinema, thereby accurately monitoring the opening of cinemas under the public health protection policy in the postepidemic era.

This study will analyze the impact of public health protection policies on the opening of cinemas in the postepidemic era. At the same time, the advantages of big data technology in monitoring the opening of cinemas will be fully analyzed. In the process of analyzing the performance of the intelligent monitoring platform based on big data technology, the statistical parameters of relative error and linear correlation coefficient are used. This study is organized as follows. In Section 1, the impact of COVID-19 on public places such as cinemas is analyzed, and the deficiencies of traditional monitoring platforms in monitoring the opening of cinemas after the transformation of cinemas in the postepidemic era are expounded. The research status of platforms monitoring the opening of cinemas is presented in Section 2.  Section 3 presents the established monitoring platform for the opening of cinemas based on big data technology and explains the relevant theoretical background.  Section 4 analyzes the feasibility and performance of big data technology in monitoring the opening of cinemas.  Section 5 summarizes the content of the study.

## 2. Related Work

COVID-19 has brought a severe impact on the global economy and people's lives. With the epidemic under control, many researchers studied the impact of the virus and epidemic prevention and control policies on the economy and life since the epidemic outbreak. As COVID-19 raged around the world, Feng et al. [11] analyzed the relationship between epidemic prevention and control and economic development. They constructed a measure of the effectiveness of pandemic containment and analyzed the relationship between epidemic prevention and control policies and GDP growth in multiple countries based on the constructed measure. The results of the analysis showed that to control the epidemic, the economic development of most countries has been negatively affected. In addition, Alkandari et al. [12] analyzed the impact of COVID-19 on people's lives. By reviewing recent research results, this paper analyzed the impact of the epidemic on people's lives from the perspective of mental health and analyzed the reasons for this impact. Then, based on the analysis results, corresponding measures are proposed to improve people's quality of life under the public health prevention and control policy. Under the influence of the epidemic, public places such as movie theaters are inevitably under control. Then, to explore the impact of public health prevention and control policies on the box office revenue of cinemas, Kim [13] proposed a nested logit model. Based on the proposed model, this paper analyzes the impact of epidemic prevention and control policies in public places on the box office of cinemas. Subsequently, Valck and Damiens [14] analyzed the impact of epidemic spread and public health protection policies on public activities involved in the film industry. Based on the analysis results, this paper described the development opportunities of the industry under epidemic prevention and control. Under the epidemic prevention and control policy, traditional box office monitoring methods cannot fully reflect the opening of movie theaters. Consider the application of big data technology in enterprises, explore how to improve the competitiveness of small and medium-sized enterprises in epidemic prevention and control based on big data technology, and use big data technology to improve the business operation ability of epidemic prevention and control enterprises [15, 16]. Although big data technology has been applied in other fields in the postepidemic era, there are still gaps in monitoring the opening of cinemas. Therefore, this study makes full use of a large amount of data generated by the cinema platform, such as platform ticket data and public place code data, and exerts the feature extraction ability of big data technology, trying to develop a big data monitoring platform to monitor the opening of cinemas.

## 3. Monitoring Platform for the Opening of Cinemas in the Postepidemic Era

### 3.1. The Importance of Big Data Technology in Improving the Monitoring Platform of Cinemas

The epidemic has brought an unprecedented impact on the business model of public places such as cinemas. Although the spread of the epidemic has been effectively contained through a series of measures, in the postepidemic era, public places such as cinemas are constrained by public health protection policies, and their regular movie screening revenue has shrunk significantly compared to before. Under the influence of epidemic prevention and control policies in the postepidemic era, cinemas have innovated and transformed their business models to increase revenue. A variety of entertainment items have been added to the transformed cinemas, while traditional cinema opening monitoring platforms mainly monitor traditional indicators such as movie ticket sales data and attendance rates, which have limitations in monitoring the flow of people in cinemas. Due to the large time uncertainty of the flow of people in the cinema and the consumption behavior of these mobile people sometimes cannot be accurately recorded, the traditional monitoring platform cannot accurately reflect the actual opening of the cinema. The emergence of public place codes in the postepidemic era has made people's access to public places traceable. The place codes in cinemas will also generate a large amount of code scanning data when people enter and exit the cinema. Therefore, this study introduced big data technology to improve the monitoring accuracy of cinema openings. The monitoring platform based on big data technology has the function of the traditional monitoring platform to record the sales of movie tickets. Moreover, the intelligent monitoring platform can obtain the data of people flow in the cinema by analyzing the code scanning data of the public place code.

### 3.2. Big Data Technology-Based Monitoring Platform for the Opening of Cinemas

Based on the sales data of e-tickets generated by the Internet platform, as well as the scan code data information of public places under epidemic prevention and control, big data technology can give full play to its data mining capabilities and extract feature information that characterizes the opening of cinemas from these data. Because the collected big data information contains not only picture information but also sequence information that changes with time, while CNN and LSTM are more suitable for extracting the feature information contained in these two kinds of data, this study adopts the CNN-LSTM hybrid network to extract the feature information contained in the big data that reflects the opening of cinemas. CNN and LSTM are two commonly used network structures in deep learning (a branch of big data technology) [17, 18]. Among them, CNN can extract the feature information contained in the images collected in the cinema [19], and LSTM can extract the time-related feature information contained in the time series data collected by the Internet [20]. The cinema opening monitoring platform based on the CNN-LSTM hybrid network is shown in Figure 1.

As can be seen from Figure 1, the established intelligent monitoring platform consists of two parts: the data acquisition system and the deep learning framework. The data collection system can collect data related to movie viewings, such as ticket sales data from online platforms and offline sales front desks of cinemas, and attendance data for each movie screening. In addition, the data collection system can also collect data on the flow of people in the cinema, such as code scanning data in public places and picture data reflecting the flow of people in cinema image systems. Based on the data obtained by the data acquisition system, CNN-LSTM can extract feature information that reflects the opening of cinemas contained in the data and output indicators representing the opening of cinemas in its network output layer. Based on the indicators in the output layer of CNN-LSTM, the opening of the cinema can be monitored.

In the following, a brief introduction to the CNN-LSTM framework adopted in this study is given.

The two network structures, CNN and LSTM, are good at feature extraction in different ways. For CNN, it is proposed to improve image recognition performance. Moreover, its weight-sharing feature greatly reduces the number of trainable parameters in the network, thereby reducing the complexity of the network. In addition, the translation invariance of CNN enables it to fully extract the local correlation feature information of adjacent locations in the input. Therefore, in the established intelligent monitoring platform, CNN can fully analyze the feature information contained in the collected cinema image data. On the other hand, LSTM is obtained by improving RNN, which alleviates the long-term memory decay problem of RNN. Therefore, LSTM has good performance when dealing with long sequence correlation problems. According to the above analysis of CNN and LSTM, although CNN can extract the image feature information contained in the collected data since the collected data also contains time-related sequence information, it is not enough to use CNN alone. Therefore, LSTM is added to the intelligent monitoring platform to extract the time-correlated feature information contained in the big data, thereby improving the monitoring accuracy of the cinema open monitoring platform.

In the CNN-LSTM framework, the forward propagation formula of CNN is

(1) $$\begin{array}{c} a^{l}=f\left(z^{l}\right)=f\left(W^{l}*a^{l-1}+b^{l}\right), \end{array}$$

where *W*^*l*^ and *b*^*l*^ represent the weights and biases of the *l*th layer, respectively; *z*^*l*^ and *a*^*l*^ represent the input and output of the *l*th layer, respectively; and *f* represents the activation function of the network layer. To alleviate the abnormal gradient problem in network information propagation, this study uses the ReLU function as the activation function in convolutional layers [21], where the mathematical expression of the ReLU function is

(2) ReLUx=max0,x.

It can be seen from equation (2) that the output value of ReLU can be greater than 1, which can promote the propagation of gradient information. In addition, ^*∗*^ represents a convolution operation on weights and network layer inputs, and the operating principle of convolution operation in convolutional layers is presented in Figure 2. As can be seen from Figure 2, the convolution operation is actually the sum of the elementwise products between the weights and the input of the convolutional layer. Moreover, Figure 2 indicates that the convolutional layers can extract locally relevant information within the convolution kernel size range.

For LSTM, it adds three gated control structures compared to the traditional RNN: forgetting gate, input gate, and output gate [22]. The structure diagram of LSTM is shown in Figure 3.

The mathematical expressions of the three gated structures are

(3) $$\begin{array}{c} f_{t}=\sigma \left(W_{f}\cdot x_{t}+W_{f}\cdot h_{t-1}+b_{f}\right), \end{array}$$

(4) $$\begin{array}{c} i_{t}=\sigma \left(W_{i}\cdot x_{t}+W_{i}\cdot h_{t-1}+b_{i}\right), \end{array}$$

(5) $$\begin{array}{c} o_{t}=\sigma \left(W_{o}\cdot x_{t}+W_{o}\cdot h_{t-1}+b_{o}\right). \end{array}$$

where *W*_*f*_ and *b*_*f*_ represent the weights and biases of the forgetting gate, respectively; *f*_*t*_, *i*_*t*_, and *o*_*t*_ represent the output of three control gates; and *σ* represents the sigmoid activation function.

The outputs of the three control gates can be obtained through the nonlinear calculation of equations (3)–(5). At this time, the state and output of the LSTM unit can be further calculated, and the calculation formula is

(6) $$\begin{array}{c} C_{t}=f_{t}\circ C_{t-1}+i_{t}\cdot C_{t-1}^{\prime }, \end{array}$$

(7) ht=ot∘ReLUCt.

Equations (6) and (7) are the state and output of the LSTM unit, respectively, where ◦ represents the elementwise product operation.

The above is a brief description of CNN and LSTM. With the feature information extracted by CNN and LSTM, it is also necessary to establish a mapping relationship between the feature information and the cinema opening indicators. In this study, to improve the generalization performance of the network, fully connected layers are adopted to realize this mapping relationship. The expression of the fully connected layer is

(8) $$\begin{array}{c} a^{l}=f\left(z^{l}\right)=f\left(W^{l}a^{l-1}+b^{l}\right). \end{array}$$

Since multiple indicators are required to quantify the opening of cinemas, the softmax activation function is used in the output layer of the CNN-LSTM framework, and its expression is

(9) $$\begin{array}{c} a^{l}=\text{soft}\max\left(z^{l}\right)=\frac{\exp\left(z_{i}^{l}\right)}{\sum_{i=1}^{K}\exp\left(z_{i}^{l}\right)}, \end{array}$$

where *K* represents the number of quantitative indicators. As indicated in equation (9), all output values of the softmax function are in the range (0, 1), which can improve the training efficiency of the network.

With a large amount of data representing the opening of cinemas, in the process of training CNN-LSTM, a loss function needs to be calculated to evaluate the training progress of CNN-LSTM. Since the prediction of cinema opening indicators is a regression problem, the loss function based on mean square error is adopted in this study, and its expression is

(10) $$\begin{array}{c} \text{Loss}=\frac{1}{S}\sum_{s=1}^{S}\sum_{i=1}^{K}{\left(y_{i}^{\text{pre}}-y_{i}^{\text{real}}\right)}^{2}, \end{array}$$

where *S* represents the number of samples participating in the network training and *y*^pre^ and *y*^real^ represent the predicted value of CNN-LSTM and the real value of the evaluation index, respectively. According to equation (10), Loss can represent the comprehensive error of multiple indicators in all samples.

## 4. Results of Analysis and Discussion

In the postepidemic era, from the perspective of public health, this study establishes an intelligent monitoring platform based on CNN-LSTM to monitor the opening of cinemas. The established intelligent monitoring platform takes into account the characteristics of cinemas after the transformation of the postepidemic era and also considers the health code data under the public health protection policy as big data information. To explore the monitoring accuracy of the intelligent monitoring platform established in this study on the opening of cinemas in the postepidemic era, we conduct a case study in this section. Since big data technology requires a large amount of data as support, we take 5,000 cinemas as the research object and use a large amount of data from these cinemas to train CNN-LSTM. The data collected from these cinemas include the picture data of the cinema image system, the online and offline ticket purchase data, and the scan code data of the public place code. To evaluate the opening of cinemas, three indicators such as attendance rate, cinema revenue, and people flow are selected as the output of the intelligent monitoring platform. Since the three quantitative indicators have different dimensions, to improve the performance of the intelligent monitoring platform, the three indicators are all normalized. The normalization processing method used in this study is the 0-1 normalization method, and its expression is

(11) $$\begin{array}{c} \text{Norm}\left(y\right)=\frac{y-\min\left(y\right)}{\max\left(y\right)-\min\left(y\right)}. \end{array}$$

Through 0-1 normalization, the value ranges of the three quantitative indicators are unified as (0, 1); then, the distribution of the quantitative indicators is closer to the data distribution of the CNN-LSTM output layer, which is beneficial to improving the training efficiency of the network. Note that to maintain the availability of the evaluation indicators, it is also necessary to denormalize the normalized indicators and finally use them as the output of the intelligent monitoring platform.

With the processed data, the effectiveness of CNN-LSTM in predicting cinema opening indicators can be explored. Meanwhile, in this section, the necessity of adding LSTM to the intelligent monitoring platform is evaluated by comparing CNN-LSTM and the traditional CNN. In the process of evaluating the prediction performance of the network, the relative error is adopted to evaluate the difference between the predicted and real results. The formula for calculating the relative error is

(12) $$\begin{array}{c} \text{RE}=\frac{\text{abs}\left(y^{\text{pre}}-y^{\text{real}}\right)}{y^{\text{real}}}, \end{array}$$

where abs is the operation for calculating absolute values. With a CNN structure alone, the average relative error distributions between the predicted and real indicators are shown in Figure 4. In Figure 4, “1,” “2,” and “3” of the horizontal axis represent the three indicators of attendance, cinema, and people flow, respectively. As can be seen from Figure 4, the average relative error between the predicted and real values of the cinema revenue indicator is relatively large, reaching 3.12%. The average relative errors of the predicted and real values of the other two indicators, attendance and people flow, are 1.89% and 2.31%, respectively. Although the average relative error of the three indicators is less than 5%, the average relative error of the cinema revenue indicator exceeds 3%, so there is still a gap for improvement.

To present the difference between the CNN-LSTM structure and CNN alone in predicting cinema opening indicators, the average relative error between the three indicators predicted by CNN-LSTM and the real values is calculated. The average relative errors between the predicted and real values of the three indicators are shown in Figure 5. It can be seen from Figure 5 that the average relative error levels corresponding to the three indicators are relatively close. Comparing Figures 4 and 5, it can be seen that compared with CNN, CNN-LSTM has improved the prediction accuracy of the three indicators, especially for the cinema revenue indicator, the average relative error reached 1.99%. At the same time, the other two indicators have also been improved to a certain extent, which are 1.55% and 1.71%. The reasons for the superiority of CNN-LSTM over CNN in the prediction of the three indicators can be explained as follows. The three indicators, especially the cinema revenue data, have time-related characteristics, so adding LSTM, which is good at extracting time-correlated features, to the intelligent monitoring platform is beneficial to improving the monitoring accuracy of cinema opening indicators.

Figure 5 indicates that the average relative errors for the three cinema opening indicators are all within 2%. However, the cinema revenue indicator is very close to 2%. Since revenue indicators are very critical in reflecting the opening of cinemas, to more intuitively present the prediction performance of the intelligent monitoring platform for cinema revenue indicators, Figure 6 shows the relative error between the predicted and real values corresponding to the 15 samples. As can be seen from Figure 6, the relative error between the predicted and real values of the cinema revenue indicator is basically within 2%, and only the relative error corresponding to the two samples is slightly greater than 2%, but the relative error of these two samples is still within 2.5. Therefore, the prediction results of the cinema revenue indicator indicate that the intelligent monitoring platform based on CNN-LSTM is feasible for monitoring the opening of cinemas.

To further analyze the performance of the intelligent monitoring platform based on CNN-LSTM, the correlation between the predicted cinema attendance and the real cinema attendance is compared.  Figure 7 presents the predicted and real cinema attendance results for 15 samples. Among them, the green area corresponding to A represents the real cinema attendance, and the blue area corresponding to B represents the cinema attendance predicted by the intelligent monitoring platform. It can be seen from Figure 7 that the average of the predicted and real cinema attendance rates are 0.7087 and 0.6921, respectively, and the predicted and real attendance data distributions corresponding to 15 samples are very close. Since the attendance rate close to 0.7 is very different from the attendance rate close to 1 in the nonepidemic period, the prediction results show that the intelligent monitoring platform based on CNN-LSTM can effectively extract the feature information that characterizes the public health protection policy, thereby making the predicted value of the attendance rate that is very close to the real value under the epidemic background. Therefore, the prediction results of the cinema attendance indicator further indicate that the established intelligent monitoring platform has good accuracy in monitoring the cinema opening indicators.

For the human flow indicator, this study uses statistical analysis methods to analyze the predictive performance of the intelligent monitoring platform.  Figure 8 shows the correlation relationship between the people flow predicted by the intelligent monitoring platform and the real people flow. The two coordinates of the data points in Figure 8 represent the real and predicted people flow. As can be seen from Figure 8, the data points are basically close to the line *y* = *x*. In addition, the calculation results of linear correlation show that the linear correlation coefficient between predicted and real people flow is 0.9802. As indicated in reference [23], a linear correlation coefficient greater than 0.95 indicates a strong linear correlation between the predicted and real results. So, based on the distribution of data points and the calculation of the linear correlation coefficient, there is a strong linear correlation between the predicted and real people flow. Therefore, the calculation results of linear correlation further validate that the established intelligent monitoring platform can accurately predict the opening of cinemas from the perspective of statistical analysis.

## 5. Conclusions

COVID-19 has brought unprecedented changes to people's lives. The easy-to-spread nature of the virus makes the public health protection system face a severe test. Although the vaccination of vaccines and the improvement of medical facilities have kept the epidemic at a generally controllable level, in the postepidemic era, there are still a series of restrictions on activities in public places. Under the public health and epidemic protection policy in the postepidemic era, cinemas have to transform to maintain normal income levels. Due to the impact of epidemic prevention and control measures, the business model of cinemas has changed. Conventional monitoring platforms usually focus on monitoring box office changes but cannot accurately monitor the opening of transformed cinemas. To overcome the shortcomings of traditional monitoring platforms, this study introduced big data technology to analyze the feature information contained in the numerous data collected from cinemas and establishes an intelligent monitoring platform based on CNN-LSTM to monitor the opening of cinemas.

When analyzing the data, the intelligent monitoring platform based on CNN-LSTM not only considers the box office data collected by cinemas under the traditional business model but also considers the impact of public health and epidemic protection policies on the opening of cinemas in the postepidemic era. In the intelligent monitoring platform, the framework composed of CNN and LSTM can extract the picture information collected from the cinema imaging system and the feature information contained in the box office data collected from the cinema sales platform and can also analyze the characteristic information of people flow contained in public place codes under epidemic prevention and control. Based on the extracted feature information, the intelligent monitoring platform can output quantitative indicators that characterize the opening of the cinema. This study analyzes the performance of the established intelligent monitoring platform in predicting the opening of cinemas through a case study. The research results show that the CNN-LSTM-based framework has better prediction performance than the CNN framework alone, especially for the prediction of cinema revenue indicators with time-related characteristics. In addition, most of the relative errors of the intelligent monitoring platform's predictions on the three indicators such as attendance, cinema revenue, and people flow are less than 2%, which indicates that the predicted and real cinema opening indicators are in good agreement. Besides, the statistical analysis results show that the linear correlation coefficient between the predicted and real people flow is 0.9802, which indicates that there is a strong linear correlation between the people flow predicted by the intelligent monitoring platform and the real result. Therefore, from the perspectives of relative error and statistical analysis, it is confirmed that the established intelligent monitoring platform has good performance in monitoring the opening of cinemas.

## Figures and Tables

**Figure 1:** Intelligent cinema opening monitoring platform based on CNN-LSTM.

**Figure 2:** Specific process of the convolution operation.

**Figure 3:** The structure of the LSTM cell.

**Figure 4:** Average relative error distributions between the predicted and real indicators under the CNN structure.

**Figure 5:** Average relative error distributions between the predicted and real indicators under the CNN-LSTM structure.

**Figure 6:** Relative error distributions between the predicted and real cinema revenue indicators corresponding to the 15 samples.

**Figure 7:** The distribution of the predicted and real cinema attendance rates corresponding to 15 samples.

**Figure 8:** Correlation relationship between the predicted and real people flows.

## Data Availability

The data set can be accessed through the corresponding author upon request.
